# A Rehabilitation Model Conducive to Postoperative Recovery of Endometrial Cancer Patients after Laparoscopy

**DOI:** 10.1155/2022/9910841

**Published:** 2022-09-02

**Authors:** Li Yang, Feng Han

**Affiliations:** ^1^Department of Pediatric Urology, Shengjing Hospital of China Medical University, Shenyang, Liaoning 110004, China; ^2^Department of Obstetrics and Gynecology, Shengjing Hospital of China Medical University, Shenyang, Liaoning 110004, China

## Abstract

Although collaborative care is increasingly being implemented in the treatment of various diseases, there are currently no related studies on its effects in endometrial cancer patients after laparoscopic treatment. Thus, this study is aimed at investigating the significance of an integrated medical and nursing care model for women with gynecologic malignant tumors who underwent laparoscopic treatment. The patients were randomly divided into a medical-nursing integrated nursing group (study group) and a general nursing group (control group). Their serum carbohydrate antigen 19-9 (CA19-9), human epididymal protein 4 (HE4), CA15-3, and CA125 levels were measured at admission, 7 and 15 days after admission, and 30 days after discharge. Their first postoperative flatulence time, eating time, and hospitalization duration were recorded, and the self-rating anxiety scale (SAS) and self-rating depression scale (SDS) were used to evaluate the psychological state of the patients. A questionnaire survey was also used to evaluate their satisfaction with nursing. Adverse events within 2 years of follow-up were recorded. The results showed that the clinical performance of the study group was significantly better than that of the control group. Further, the study group demonstrated significantly lower serum tumor marker levels, SAS score, SDS score, and incidence of adverse events at 7 and 15 days after admission and 30 days after discharge and higher nursing satisfaction than the control group. Thus, the collaborative nursing mode might be more conducive to the recovery of women who have underwent laparoscopic treatment for gynecologic malignant tumors than normal routine nursing.

## 1. Introduction

Endometrial cancer is the most common gynecological malignancy with a growing incidence [1]. It led to approximately 320,000 new cases and 76,000 deaths in 2012 [2]. According to statistics, it is the sixth most common cancer worldwide and the 14th leading cause of cancer death in women [3]. At present, hysterectomy and the removal of the fallopian tubes and ovaries are considered the standard treatment for women with endometrial cancer, while radiotherapy and chemotherapy are regarded as common auxiliary treatments [4]. Ben-Hur and Phipps described the first laparoscopic-assisted vaginal hysterectomy in 1989 [5]. With the advancement in cancer research, minimally invasive treatment such as laparoscopic surgery has been increasingly used and started to replace the traditional open surgery in endometrial cancer treatment [6]. However, it was recently reported that the incidence of laparoscopic-associated adverse events, such as lymphedema, neuropathy, and wound infection rates, for endometrial cancer was quite high, at ~21%, and might even reach 33% in some settings [7]. Therefore, postoperative care for endometrial cancer patients is particularly important to timely identify and treat complications and enhance their recovery.

The postoperative recovery of patients was found to be closely associated with the methods and mode of nursing. Collaborative care is a complex intervention for depression developed in the United States. Specifically, collaborative care has advantages like combined multiprofessional approaches to patient care, structured management plans, scheduled patient follow-up, and enhanced interprofessional communication [8]. The collaborative care model has been recognized as pivotal in improving the management of various chronic diseases [9]. In addition, collaborative care has been shown to improve the short- and long-term depression outcomes more effectively than standard care. Further, incremental evidence shows that collaborative care can improve the prognosis and recovery of patients with long-term chronic diseases such as diabetes [10], significantly reduce the length of hospital stay of patients with gastrointestinal cancer, and improve patients' quality of life [11]. Thus, based on existing literature, we believe that collaborative care would also benefit patients with reproductive system cancer.

However, there are currently no studies on the effects of integrated nursing involving doctors and nurses under a collaborative care model for the laparoscopic treatment of endometrial cancer patients. To fill this gap, we performed this study to compare the effects of collaborative care versus general care on women who underwent laparoscopic treatment for endometrial cancer to provide an effective theoretical basis for potentially improving the treatment and outcomes of endometrial cancer patients.

## 2. Materials and Methods

### 2.1. Study Subjects

The data of 1144 patients with endometrial cancer who underwent laparoscopic treatment in our hospital from March 2018 to February 2021 were collected. Inclusion criteria are as follows: (1) patients diagnosed with endometrial cancer based on comprehensive clinical diagnosis and treated by laparoscopy; (2) surgery naïve patients, older than 18 years old; (3) could communicate normally and complete the study survey in oral or written form; and (4) patients and their families were informed and signed the informed consent form, agreeing to participate in the study. Exclusion criteria are as follows: (1) patients with other malignant tumors; (2) presence of severe liver and kidney function damage, cardiovascular disease, or other serious organ and tissue diseases; (3) patients with severe mental illness, severe cognitive impairment, or language problems; and (4) contraindications to study treatment. After admission, the patients were divided into a study group (*n* = 572) and a control group (*n* = 572) according to different nursing methods at the treating physician's discretion. The study group adopted integrated nursing with doctors and nurses based on a collaborative care model, mainly including (1) establishment of a consultation group based on the collaborative care model; (2) primary evaluation of admitted patients by the consultation group; (3) ward round by the consultation group; (4) patient care during admission and guidance by the consultation group; and (5) provided psychological care to the patients. Routine nursing was applied in the control group, mainly comprising examination on admission, guidance on diet, exercise and drugs after admission, and general health assessment and guidance. The general data of all patients were recorded, including age, gender, height, weight, education, age of onset, disease duration, tumor stage, pathological type, past medical history, complications, and follow-up time. Informed consent was obtained from all patients, and this study was approved by the Ethics Committee of Shengjing Hospital of China Medical University (No. 2022PS147K).

### 2.2. Detection of Serum Tumor Markers

All patients were drawn 4 ml of peripheral venous blood on an empty stomach at admission, 7 and 15 days after admission, and 30 days after discharge. After standing for 20 min, the blood was centrifuged at 3000 r/min for 10 min. Then, the supernatant was aspirated and stored at -20°C. The level of carbohydrate antigen 19-9 (CA19-9), human epididymis protein 4 (HE4), carbohydrate antigen 15-3 (CA153), and carbohydrate antigen 125 (CA125) in serum was measured with an automatic biochemical analyzer (Mindray, China).

### 2.3. Evaluation of Psychological Status

All patients were graded using a self-rating anxiety scale (SAS) and self-rating depression scale (SDS) before nursing, 7 and 15 days after nursing, and 30 days after discharge. Then, according to the score, the psychological status of patients in the two groups before and after nursing was evaluated.

#### 2.3.1. SAS Score

Each item was graded on a level of 1-4 according to the sensation in the last week, and the cumulative score of each item was regarded as the total SAS score. The SAS standard score was defined as follows: less than 50, no anxiety; 50-59, mild anxiety; 60-69, moderate anxiety; and greater than 70, severe anxiety [12].

#### 2.3.2. SDS Score

It ranged from 1 to 4 levels. The score for each item was then calculated to obtain the overall score, which was classified as follows: less than 50, no depression; 50-59, mild depression; 60-69, moderate or high depression; and greater than 70, severe depression [12]. The criterion score = overall score^∗^1.25.

### 2.4. Evaluation of Clinical Indicators during Hospitalization

To determine the significance of the collaborative nursing mode during hospitalization, the following postoperative recovery-associated indicators were recorded and assessed: time taken to first postoperative exhaust, time taken to first postoperative food-taking, and overall hospital stay (from admission to discharge).

### 2.5. Evaluation of Satisfaction with Care

A self-made satisfaction questionnaire (total points, 100) was used to assess the two groups' satisfaction with nursing care. The scoring criteria were as follows: unsatisfactory, 0-59 points; satisfactory, 60-89 points; and very satisfactory, 90-100 points.

### 2.6. Postoperative Follow-Up

Patients in both groups were followed up for 2 years after surgery, and adverse events or complications during follow-up were recorded.

### 2.7. Statistical Analysis

SPSS 25.0 software was used for data analysis. The measurement data with normal distribution was expressed as mean ± standard deviation (SD). The mean of multiple groups was compared by one-way ANOVA, and pairwise comparison was performed by *t*-test. The categorical data was described by frequency (*n*) and percentage (%), and the difference between groups was assessed by using chi-square test or Fischer's exact test. *P* < 0.05 indicated statistical significance.

## 3. Results

### 3.1. General Information of Patients

The basic characteristics of the study and groups are shown in Table 1. The mean age of patients in the two groups was around 61 years (study vs. control group, 61.00 ± 9.54 vs. 61.69 ± 6.86), and the age of onset was around 55 years. There was a relatively higher proportion of patients for tumor stage 1. There were no significant differences between the two groups in gender, age, height, weight, histological classification, past medical history, and complications (Table 1), indicating the two groups of patients were comparable.

### 3.2. Collaborative Care Effectively Reduced the Level of Serum Tumor Markers at Different Periods and Improved the Mood of Patients

The levels of serum tumor markers, CA19-9, HE4, CA153, and CA125, were determined at the indicated time. The results showed no significant difference in serum tumor marker levels at admission between the two groups. However, after admission, the level of serum tumor markers of patients in both groups gradually decreased, with patients in the study group demonstrating a significantly greater decrease than the control group at 7 and 15 days after admission and 30 days after admission (Figure 1(a)). Similarly, the two groups had no significant difference in SAS and SDS scores at admission, but after admission, a decrease in SAS and SDS scores was observed in both groups. We observed that the SAS and SDS scores of patients in the study group were significantly lower than those of the control group at 7 and 15 days of admission and 30 days of admission (Figure 1(b)). The above results suggested that collaborative care was more effective than routine care in the recovery of patients with endometrial cancer.

### 3.3. Collaborative Care Can Effectively Reduce Relevant Clinical Indicators of Patients during Hospitalization

The relevant clinical indicators during hospitalization were compared between the two groups. The results showed a significantly shortened time to first postoperative exhaust (4.52 ± 1.10 days), postoperative food-taking (5.46 ± 1.70 days), and hospital stay (24.85 ± 4.42 days) in the study group compared with the control group (Table 2).

### 3.4. Collaborative Care Can Improve Patients' Satisfaction with Nursing

The satisfaction rate of nursing care in the two groups was also evaluated. The results indicated that the satisfaction rate of patients with nursing care in the study group was mostly “very satisfied” (*n* = 347), while that in the control group was mostly “satisfied” (*n* = 240). In addition, there were 19 “dissatisfied” cases with nursing care in the study group, while in the control group, the number of “dissatisfied” cases was 99. Overall, the patients' satisfaction with nursing care in the study group was as high as 96.67%, which was significantly higher than that in the control group (82.69%) (Table 3).

### 3.5. Collaborative Care Can Significantly Reduce the Incidence of Postoperative Adverse Events in Patients

After 2 years of follow-up in both groups, adverse events and complications were recorded. The results revealed that the main complications of patients in the study group included fever, lymphocele, and intestinal obstruction. The control group contained 13 cases with urinary retention, 13 cases with pulmonary embolism, and 11 cases with ureteral fistula, while patients in the study group had no such complications. In addition, there was only one case of poor healing of vaginal stump and brain obstruction in the study group, while the control group had more than 10 cases of complications. The above result displayed that patients in the study group had a distinctly lower incidence of adverse events and complications than those in the control group (Table 4).

## 4. Discussion

In this study, using a large cohort of 1144 patients, we investigated the significance of a rehabilitation model via collaborative nursing consisting of doctors and nurses for endometrial cancer patients after laparoscopy compared with routine nursing care. The results showed that collaborative care was associated with a significantly faster reduction in serum tumor marker, an improved mood of patients, faster in-hospital postoperative recovery, greater satisfaction with the nursing offered, and reduced risk of postoperative adverse events. An important strength of this study was that the patients from both groups were well balanced in terms of age, education level, tumor stage, histological classification, past medical histories, and major complications such as hemorrhage, infection, and intestinal problems, which might have otherwise significantly affected the recovery of the patients, thereby biased this study's important indicators such as changes in tumor markers and in-hospital postoperative recovery.

Collaborative care interventions were designed to provide more individualized support and care coordination to patients across the continuum of care. For example, in such settings, dedicated health care professionals are able to timely assess, treat, and monitor patient conditions throughout the whole hospitalization period and even after discharge. Collaborative care interventions have been confirmed to be effective in chronic disease care [13, 14]. A recent meta-analysis of 37 collaborative care intervention studies on 12,355 patients found that depression was improved at 6-month follow-up, and long-term benefits up to 5 years were also observed [15]. Besides, Dwight-Johnson et al. reported significantly reduced depression and good prognosis in samples of patients with breast and cervical cancer after applying collaborative care approaches [16]. Similarly, this study found that collaborative care intervention was superior to routine care.

Collaborative care enhances the interactions between patients and healthcare professionals via the identification of multiple physical, psychological, social, and spiritual needs of the patients and the implementation of evidence-based supportive care interventions flexibly and responsively in the context of a collaborative multidisciplinary approach to care, to achieve optimal health outcomes for the patients [17, 18]. Thus, based on this interactive guidance and continuous support, the patients in the study group demonstrated faster time to exhaust and oral food intake and shorter hospital stays. Further, these also led to a significantly greater degree of satisfaction in the study group compared with this control group (study vs. control group, 96.67% vs. 82.69%), especially considering that the patients had more psychological support and guidance by the treating hospital staff members. These findings also indicate that collaborative care-based services could be of high value in regulating patients' physical and mental states, especially for those with cancer.

We also observed that the study group had a significantly lower risk of postoperative complications such as poor healing of wounds, urinary retention, and lung infections, among others. The major sequelae after endometrial cancer surgery include symptoms similar to menopause as well as sexual dysfunction [19]. Although some studies have pointed out that laparoscopic surgery can improve the above adverse effects compared to open surgery [20], some other studies have also shown that there is some consequential amount of abdominal bleeding despite laparoscopic surgery [20], and the incidence of bladder injury [21] and vascular injury reaches 1% [22]. Interestingly, in this study, we found that collaborative care could significantly reduce the incidence of symptoms such as blood loss, bladder injury, vascular injury, and ureteral injury. We believe that the main reasons could be as follows. First, the interventions (i.e., changing of dressings and vital sign assessment) for patients with conventional care are mainly performed by students or nurses alone, while the managing physicians are mainly responsible for major systemic treatment, and there might be a lack of timely and direct communication between them resulting in lack of adequate attention to factors that might have potentially led to these complications [23]. The collaborative care-based nursing can effectively avoid the above-mentioned shortcomings as it integrates the medical and nursing personnel to form an intervention team, which improves the standardization and systematization of treatment and results in better treatment outcomes for the patients [24].

Further, the adoption of multidisciplinary team-based nursing care not only led to decreased complications but might have also directly affected the reduction of serum tumor levels, SAS score, and SDS score. Postoperative complications can be described as a deviation from the normal postoperative course and can be classified in terms of severity or infective/noninfective etiology [25]. Although the patients were well balanced in several demographics and clinical characteristics, the significantly faster decrease in serum tumor markers needs further investigation. We hypothesize that there may be a relationship between patients' tumor markers, other biochemistry markers, complications, and immunity. Patients in the study group received greater attention and care by an intervention team, which led to timely identification of issues in biochemistry markers, such as white blood cell, neutrophil and hemoglobin counts, and levels of C-reactive protein (CRP), albumin, and interleukin-6 (IL-6), and therefore possibly faster treatment compared with the control group. Thus, lesser aggravation in the condition of the patients from the study group might have contributed to a faster decrease in tumor markers and lesser interference with other biochemical markers compared with the control group. In addition, the better SAS and SDS scores observed in the study could be attributed to the lower physical stress and emotional and financial burden compared to the control group.

Despite the interesting findings observed in this study, there were several limitations worth mentioning. First, this was a single-center retrospective study; therefore, the presence of some bias might have been inevitable. However, considering that many of the important characteristics between the two groups of patients were well-balanced (Table 1), we believe this might not have significantly affected the overall study results. Second, the association between serum tumor markers and other serological markers (i.e., inflammatory and nutritional) was not assessed; therefore, the faster decrease in tumor marker levels in the study group requires further investigations. Lastly, longer follow-up might be needed to determine the possible association of collaborative care in terms of patients' survival and tumor recurrence risk compared with routine nursing.

## 5. Conclusions

In summary, compared with routine nursing, collaborative care can enhance the rehabilitation of patients with endometrial cancer and improve their psychological status and satisfaction with nursing. Moreover, collaborative care can improve the outcomes of laparoscopic treatment of endometrial cancer. The results of this study provide preliminary support for the application of collaborative care in the treatment of endometrial cancer, especially after laparoscopy, and should be further validated in larger cohort of patients with multicenter prospective clinical settings.

## Figures and Tables

**Figure 1:** Comparison of serum tumor marker level and psychological scores between the collaborative and routine care groups. (a) Serum level of CA19-9, HE4, CA153, and CA125 of the two groups at different admission periods. (b) Comparison of SAS and SDS scores of the two groups at different admission periods. ^∗^*P* < 0.05 and ^∗∗^*P* < 0.01 vs. routine care group.

**Table 1:** Basic characteristics of patients from the study and control groups.

Characteristics	Study group (*n* = 572)	Control group (*n* = 572)	*t*/*χ*^2^	*P* ^∗^
Age (years)	61.00 ± 9.54	61.69 ± 6.86	1.402	0.161
Height (cm)	158.64 ± 5.82	158.47 ± 5.70	0.488	0.626
Weight (kg)	61.66 ± 7.18	62.27 ± 5.80	1.581	0.114
Education background, *n* (%)			2.172	0.338
Elementary school	384 (67.1)	407 (71.2)		
Senior high school	127 (22.2)	112 (19.6)		
College and above	61 (10.7)	53 (9.4)		
Age of onset (years)	55.51 ± 9.54	55.21 ± 7.09	1.393	0.164
Tumor staging, *n* (%)			2.219	0.528
Stage 1	295 (51.6)	288 (50.4)		
Stage 2	96 (16.8)	95 (16.6)		
Stage 3	116 (20.2)	134 (23.4)		
Stage 4	65 (11.4)	55 (9.6)		
Histological classification, *n* (%)			1.850	0.174
Endometrioid adenocarcinoma	524 (91.6)	536 (93.7)		
Other types of cancer	48 (8.4)	36 (6.3)		
Past medical history, *n* (%)			2.386	0.122
Related cases	480 (83.9)	460 (80.4)		
Unrelated cases	92 (16.1)	112 (19.6)		
Complications, *n* (%)			2.092	0.554
Hemorrhage	340 (59.4)	329 (57.5)		
Infection	168 (29.4)	179 (31.3)		
Intestinal problems	31 (5.4)	24 (4.2)		
Other	33 (5.8)	40 (7.0)		

^∗^ *P* value vs. control group.

**Table 2:** Comparison of relevant clinical indicators during hospitalization between the two groups.

Variables	Study group (days)	Control group (days)	*t*	*P* ^∗^
Time to first postoperative exhaust time	4.52 ± 1.10	7.88 ± 1.96	35.713	<0.001
Time to first postoperative food-taking	5.46 ± 1.70	6.44 ± 1.10	11.544	<0.001
Hospital stay	24.85 ± 4.42	29.18 ± 2.60	20.163	<0.001

^∗^ *P* value vs. control group.

**Table 3:** Comparison of patients' satisfaction between the two groups.

Variables	Very satisfied, *n* (%)	Satisfied, *n* (%)	Dissatisfied, *n* (%)	Degree of satisfaction
Study group	347 (60.7)	206 (36.0)	19 (3.3)	96.67%
Control group	233 (40.7)	240 (42.0)	99 (17.3)	82.69%
*χ* ^2^				60.475
*P*				<0.001^∗^

Note: a satisfaction score of 80 or above is considered very satisfied, a score of 60 to 79 (including 60 and 79) is considered satisfied, and a score of less than 60 (exclusive) is considered unsatisfied. ^∗^*P* value vs. control group.

**Table 4:** Comparison of the incidence rate of adverse events and complications after 2-year follow-up between the two groups.

Variables	Study group, *n*	Control group, *n*	*t*/*χ*^2^	*P* ^∗^
Fever	26	85	34.730	<0.001
Lymphocele	21	61	21.019	<0.001
Intestinal obstruction	19	75	36.348	<0.001
Poor healing of vaginal stump	1	11	8.422	0.004
Poor healing of abdominal incisions	2	16	11.063	0.001
Urinary retention	0	13	13.149	<0.001
Abdominal bleeding	2	25	20.066	<0.001
Vesicovaginal fistula	3	26	18.716	<0.001
Lung infection	2	34	29.369	<0.001
Brain obstruction	1	15	12.242	<0.001
Pulmonary embolism	0	13	13.149	<0.001
Ureteral fistula	0	11	11.107	<0.001

^∗^ *P* value vs. control group.

## Data Availability

Data and material are available from the corresponding author upon reasonable request.
